# A Ferroptosis-Related Gene Signature for Predicting Survival and Immunotherapy Effect in Renal Cancer

**DOI:** 10.1155/2022/3317624

**Published:** 2022-08-17

**Authors:** Liang Tong, Zhao-fa Yin, Liang Peng, Yu-ting Li, Rong Liu, Jia-rong Cai, Le Kang

**Affiliations:** Department of Urology, Loudi Central Hospital of Hunan Province, Loudi, China

## Abstract

**Background:**

Most recently, no efficient prognostic indictor is present for kidney cancer. Thus, we aimed to build and validate a new prognostic gene signature for renal cancer patients using the Cancer Genomic Atlas (TCGA).

**Methods:**

A “time-dependent receiver operating characteristic (tROC)” curve was generated, and a log-rank test was performed to assess the performance of the biomarker in training and validation. A “ferroptosis-related gene signature” was developed. In different training and validations sets, tROC and log-rank test were used to validate the biomarker's performance.

**Results:**

In the training set with a *P* value less than 0.01 and the validation set, the “gene signature” was significantly correlated with survival. Eventually, it was found that the ferroptosis-related gene signature was directly correlated with immune score and the score of tumor mutation, suggesting its role in predicting response to immunotherapy.

**Conclusion:**

We developed and validated a “ferroptosis-related gene signature” that can be sued for patients with kidney cancer. It can also assist in facilitating the plan for treatment and risk stratification.

## 1. Introduction

Renal cancer is a dangerous type of urinary cancer [1, 2], and its incidence is increasing annually [3, 4]. As renal cancer is thought of as a very heterogeneous tumor [4] and immunotherapy is still the first-line therapy for advanced renal cancer [5], immune-linked biomarkers are regarded as a predictive indicator of renal cancer [6, 7]. The diagnosis and management of renal cell carcinoma have changed remarkably rapidly. Although the incidence of renal cell carcinoma has been increasing, survival has improved substantially. Nevertheless, nowadays, biomarkers have many shortcomings and drawbacks. First, it consists of too many genes, which is difficult to identify [7, 8]. Second, the detailed mechanisms were not clarified, which still needs further study [8, 9]. So, it is very required to find a new predicting indicator for renal cancer.

Because of advances in gene sequencing technology, gene databases such as “The Cancer Genome Atlas (TCGA) [10] and Gene Expression Omnibus (GEO)” have become important reference sources. To process such large amounts of data, a variety of bioinformatics tools have been used, including “weighted gene coexpression network analysis (WGCNA) [11], cell-type identification by estimating relative subsets of RNA transcripts (CYBERSORT) [12], gene set enrichment analysis (GSEA), and least absolute shrinkage and selection operator (LASSO)” [13]. The dependability of such techniques supports the idea of employing a mix of different tools used for bioinformatics and the present databases in scientific practice [14–17].

To discover a novel immune-linked indicator for renal cancer patients, we analyzed the RNA-seq data from the cancer genome atlas by in silico approaches. We hope it will be useful for researchers and clinicians.

## 2. Materials and Methods

### 2.1. Data Acquisition

“RNA sequencing data” for 607 renal cancer cases were obtained from the “cancer genome atlas.” 516 cases of intact survival data were categorized as the training set and validation set.

### 2.2. Database for Annotation, Visualization, and Integrated Discovery (DAVID)

The Database for Annotation, Visualization and Integrated Discovery provides a comprehensive set of functional annotation tools for investigators to understand the biological meaning behind large lists of genes. DAVID (version 6.8) [18] is a website tool to annotate gene sets. It contains the “Kyoto Encyclopedia of Genes and Genomes (KEGG)” signaling pathway, “GO-BP-DIRECT, GO-CC-DIRECT,” and GO-MF-DIRECT.

### 2.3. Identification and Validation of a Ferroptosis-Gene Signature

Ferroptosis-related genes were analyzed using the “univariate Cox regression analysis” and “LASSO analyses.” The qualified genes were utilized for developing a gene signature.

The predicting ability was quantified using a risk score and assessed using receiving operating characteristics curve.

### 2.4. Gene Set Enrichment Analysis

Gene set enrichment analysis (GSEA) is a computational method that determines a priori defined set of genes statistically. Gene set enrichment analysis was performed using the GSEA software (version 4.0). The operating index was all at default.

## 3. Results

### 3.1. Identification and Validation of the Ferroptosis-Related Module

To identify a ferroptosis-related gene signature, 516 renal cancer patients with complete survival information were divided into the “training set” (*n* = 412) and “validation set” (*n* = 104). The ferroptosis-related genes were analyzed as the input of the “univariate Cox regression analysis” for the training set. 84 genes showed a significant relevance in the univariate Cox analysis. Then, the 84 genes were further analyzed using LASSO regression analysis and 27 genes showed a markedly prognostic significance (Figures 1(a) and 1(b)). Eventually, these 27 ferroptosis-related genes were used to develop a ferroptosis-related gene signature using the “multivariate Cox regression model.”

We exhibited the “risk score, survival status, and heatmap for gene expression” in a scenario where the abscissa was same to highlight the association between the ferroptosis-associated signature and the expression of genes that contained the signature and the survival of patient. The “multivariate Cox model” calculated the patient's risk score of patients which was based on the six-gene signature. If the risk scores were high, then it leads to poor survival of the patient and indicates high expression levels of the genes in the “training set” (Figure 1(c)) and the “validation set” (Figure 1(d)).

### 3.2. Evaluation of the Predictive Ability of the Ferroptosis-Associated Gene Signature

The suggested ferroptosis-related signature's predictive performance was tested in both sets. In the training and validation sets, the gene signature's 5-year AUC for predicting overall survival (OS) was 0.747 and 0.790, respectively (Figures 2(a) and 2(b)), indicating that it has a strong predictive potential for OS.

We explored the gene signature's survival value in the training and validation sets after it showed a strong prediction capacity. The risk score obtained for every patient who had gastric cancer was obtained in the TCGA cohort, and based on the median of risk scores, the patients were divided into two groups; one with high risk and one with low risks. In both sets (*P* = 0.001; Figures 2(c) and 2(d)), the low-risk group had a superior survival outcome to the high-risk group, confirming the results from the previous phase. The power of principal component analysis to discriminate was also demonstrated (Figures 2(e) and 2(f)).

### 3.3. Signaling Pathways Involved in the Ferroptosis-Related Gene Signature

The functional annotation of genes was performed by us that were connected with the ferroptosis-associated gene signature to investigate the biological processes involved with the ferroptosis-associated gene signature. Using “RNA-seq data from the TCGA cohort of patients with KIRC,” we first estimated the gene signature's association with all genes. Gene signature-related genes were chosen from 135 genes (*P* = 0.01, *R* > 0.4). Following that, the R tool “cluster profile” was used to functionally annotate these genes. Several biological processes were discovered, including the T cell leukemia signaling system and the NOD-like receptor signaling pathway (Figures 3(a)–3(d)).

### 3.4. Effect of the Ferroptosis-Related Gene Signature on Immunotherapy

We then wanted to investigate its role in response to immunotherapy. We analyzed its relationship with immune score and tumor mutation burden. Surprisingly, the established gene signature was positively correlated not only with immune score (Figure 4(a)) but also with tumor mutation burden (Figure 4(b)), suggesting its impact on immunotherapy efficacy.

## 4. Discussion

Ferroptosis is a newly form of programmed cell death that has unique biological effects on metabolism and redox biology. It is mainly caused by unrestricted lipid peroxidation and subsequent membrane damage. Ferroptotic cell death may show some morphological and biochemical characteristics as well as common changes in gene and protein levels.

We developed and validated a ferroptosis-gene signature for forecasting the lifetime and efficacy of immunotherapy for renal cancer patients. These results were very useful for the next studies. All these may lead to the advancement of novel methods for tumor therapy.

We find that the gene signature was critically linked to the immune function, underlining immune response in renal cancer. We also find multiple signaling KEGG pathways. Among them, the cell cycle was the number one in the high-risk group, supporting its role in cancer [19, 20].

This study has very good significance for renal cell carcinoma. First, we afford a novel prognostic indicator that would help the therapy of renal cell cancer. Secondly, this study found many nice signaling pathways that were effective therapeutic pathways in renal cell cancer.

## 5. Conclusion

In summary, we successfully developed and confirmed a ferroptosis-related indicator by exploring the TCGA database by in silico approaches and identified many good interesting pathways. These results could provide a basis for cancer immunotherapy.

## Figures and Tables

**Figure 1:** Identification and validation of the ferroptosis-related module.

**Figure 2:** Evaluation of the predictive ability of the ferroptosis-associated gene signature.

**Figure 3:** Signaling pathways involved in the ferroptosis-related gene signature.

**Figure 4:** Effect of the ferroptosis-related gene signature on immunotherapy.

## Data Availability

The datasets analyzed during the present study are available in the TCGA repository (https://portal.gdc.cancer.gov/).
